# Early Diagnosis and Treatment of Coronary Heart Disease with Image Features of Optical Coherence Tomography under Adaptive Segmentation Algorithm

**DOI:** 10.1155/2022/1261259

**Published:** 2022-08-08

**Authors:** Chaozhang Lin

**Affiliations:** Medical Section, Hainan Tunchang People's Hospital, Tunchang, 571600 Hainan, China

## Abstract

This research was aimed at exploring the application value of optical coherence tomography (OCT) images under adaptive segmentation algorithm in the early diagnosis of coronary heart disease (CHD). Eighty-two patients with CHD were included, who were to undergo coronary angiography (CAG) to confirm their condition. According to the diagnostic criteria of CHD in the American Coronary Artery Surgery Study (CASS), the patients were divided into the stable plaque group (41 cases) and unstable plaque group (41 cases). Besides, 20 healthy volunteers were selected as the control group, and all of them underwent OCT scans. On the basis of a fourth-order partial differential equation (PDE) and active contour (AC) model, a novel adaptive image segmentation algorithm PDE-AC was constructed and used for OCT image processing. No significant difference was found in general clinical data and serological indicators in the control group compared to the other two groups (*P* > 0.05). The lipid plaque length, degree of stenosis, and lipid pool angle, macrophages and intimal erosion, and plaque fissure in the unstable plaque group were highly greater than those in the stable plaque group. The fibrous cap thickness (FCT) was significantly thinner than that in the stable plaque group (*P* < 0.05). The diagnostic sensitivity, specificity, and accuracy of OCT under PDE-AC algorithm for CHD (91.53%, 84.08%, and 95.38%) were markedly higher than those of single OCT (83.46%, 75.11%, and 88.02%) (*P* < 0.05). In summary, OCT images under PDE-AC algorithm did better than simple OCT images in the diagnosis of CHD. Lipid plaque length, degree of stenosis, and lipid pool angle, macrophage and intimal erosion, plaque fissure, and FCT were important indicators for judging plaque stability, having the better clinical application value.

## 1. Introduction

Coronary heart disease (CHD) is a heart disease caused by coronary atherosclerosis that narrows or blocks the lumen, leading to myocardial ischemia, hypoxia, or necrosis. It is the most common organ disease caused by atherosclerosis, and males have an earlier onset than females. CHD is more common in adults over 40 years old, showing a younger trend in recent years; it is one of the major diseases threatening human health [1–3]. The clinical paradigms of CHD mainly include latent CHD, angina pectoris CHD, myocardial infarction CHD, sudden death CHD, and heart failure and arrhythmia CHD [4, 5]. The main risk of CHD is the rupture of sclerotic plaques, which induces platelet aggregation to form thrombus, resulting in acute myocardial infarction. Treatment methods include controlling factors that damage blood vessels and stopping or delaying the progression of plaques. The plaque stability is increased, and the risk of myocardial infarction can be minimized. The platelet aggregation function is inhibited, and platelet aggregation can be prevented when plaque ruptures, thereby avoiding thrombosis. If CHD is not controlled in time, angina pectoris, myocardial infarction, etc. may occur in the long-term development, which can be life-threatening in severe cases. Therefore, once many patients suffer from CHD, they will become very depressed and even maybe cannot face life positively [6]. Most people do not have any symptoms ordinarily, and their work, study, and life go as usual. But there are often signs of myocardial ischemia, such as feeling unwell of the precordium, or symptoms of fatigue. Although the symptoms are very mild, myocardial ischemia can be detected if an electrocardiogram is performed in time, so that it can be prevented as early as possible [7, 8].

As an important clinical auxiliary department, medical imaging plays an irreplaceable role for clinicians to assess the conditions. With the help of imaging, the diagnosis accuracy and efficiency of clinicians can be greatly improved. The current clinical imaging diagnostic methods for CHD mainly consists of coronary angiography (CAG), computed tomography (CT), magnetic resonance imaging (MRI), and optical coherence tomography (OCT) [9]. CAG has always been the gold standard for the diagnosis of CHD, but its diagnostic accuracy is poor, and the degree of coronary stenosis can only be roughly judged by experienced physicians [10, 11]. Coronary CT is a common method for CHD screening in the department of cardiology. It mainly develops images by injecting a contrast agent into the vein and then scans the structure of the coronary artery through CT scanning. Finally, three-dimensional reconstruction is made to get coronary images, so as to determine whether there is coronary stenosis [12]. Therefore, this is a noninvasive examination to initially determine the condition of coronary artery disease through CT scanning; but, CAG is traumatic as it needs to puncture the artery. MRI can objectively reflect myocardial perfusion and myocardial transmural degree and is the most sensitive for subendocardial myocardial lesions, but it takes a long time and is expensive [13, 14]. OCT is the latest intravascular optical scanning tomography technology used in clinical practice. It utilizes the different optical features reflected from the tissue by low-coherence near-infrared light to perform tissue analysis and imaging, and the imaging speed is fast. The greatest advantage of OCT is its high resolution. So far, it is the intravascular imaging technology with the highest resolution, which allows accurate observation of the subintimal lesions or plaques. It can be applied to identify various intravascular microstructures such as unstable plaques, stable plaques, calcification, thrombus, and dissection. Besides, OCT is expected to become an ideal method for evaluating unstable plaques in the future [15].

The quality of images is an important factor affecting the accuracy of doctors' judgment, so the enhancement of medical images is critical. The quality of the image preprocessing algorithm is directly related to the effect of subsequent image processing, like image segmentation, target recognition, and edge extraction. For high-quality digital images, it is often necessary to denoise the images, while maintaining the integrity of the original information as much as possible and removing the useless information in the signals [16]. In recent years, the partial differential equation (PDE) method derived from constrained optimization, energy minimization, and calculus of variations has been widely used in image processing. In particular, active contour (AC) has become one of the common methods of image segmentation. The PDE-AC model links the prior knowledge of the image region with the constraints of the image data, so that the AC can maintain the continuity and smoothness during the evolution process. It can well solve the issue that the initial position affects the convergence speed [17]. However, few existing studies have applied the PDE-AC algorithm to OCT image processing. In this research, patients with CHD who met the requirements were divided into two groups, and 20 healthy people were selected as the control group. The application value of OCT images under adaptive segmentation algorithm was comprehensively evaluated in the early diagnosis of CHD. Thereout, this research provided an effective solution for the clinical diagnosis and treatment of CHD.

## 2. Materials and Methods

### 2.1. Research Objects

Eighty-two CHD patients were collected as the research objects, who were scheduled to have CAG in the hospital from February 2015 to August 2020. According to the diagnostic criteria for CHD of American Coronary Artery Surgery Study (CASS), the patients were divided into the stable plaque group and unstable plaque group, with each 41 cases. In addition, 20 healthy volunteers having physical examination during the same period were included in the control group. This research had been approved by the ethics committee of the hospital. The patients and their families were informed about the research and signed the informed consent forms.

Inclusion criteria are follows: Patients had the angina pectoris CHD or myocardial infarction CHD, with typical symptoms of chest pain, having complete clinical data, and aged over 18 years old.

Exclusion criteria are as follows: (1) Patients were complicated with psychiatric diseases. (2) Patients had a stenosis rate of less than 50%. (3) Patients suffered from severe liver and kidney insufficiency. (4) Patients did not complete follow-up and lost contact midway. (5) Patients were complicated with hematological diseases. (6) Patients could not receive OCT examination for the complete coronary occlusion. (7) Patients got acute myocardial infarction.

### 2.2. Image Examination Methods

A digital subtraction system was used for performing CAG on the patients. The main projection positions included left anterior oblique+cranial position, spider position, liver position, and right anterior oblique+cranial position. After CAG, OCT scanning was performed with optical coherence tomography scanner, and 1800UI heparin was added. First, the imaging catheter was taken out and wiped with wet gauze. 2.5 mL of contrast agent was injected after the hydrophilic coating was activated. Then, system calibration was performed, and the 6F guiding catheter was inserted into the target coronary artery to lesion location. The optical display lens was adjusted to 5 mm of the proximal marker of the catheter, and the position of the 6F guiding catheter was also adjusted until smoke was emitted. The contrast medium was injected fast in a pellet manner, the light microscope was back-tested, and the system was turned off after the surgery. The acquired images were sent to the workstation for processing, and two experienced senior physicians were selected to interpret the OCT images.

### 2.3. Adaptive Image Segmentation Algorithm

In this research, the fourth-order PDE and AC model were introduced for a novel adaptive image segmentation algorithm. The energy functional of this model could be expressed as

(1) $$\begin{array}{c} F^{*}=\alpha F^{k}+\left(1-\alpha \right)F^{h}+\beta F^{i}+\lambda F^{j}. \end{array}$$

In equation (1), *F*^*k*^ denoted the global term, *F*^*h*^ denoted the local term, *F*^*i*^ was the regularization constraint term, and *F*^*j*^ was the length constraint term. *α*, 1 − *α*, *β*, and *λ* represented the global term parameter, the local term parameter, the regularization constraint term parameter, and the length constraint term parameter, respectively. Then, the edge-guided image was used to replace the original grayscale image in the AC model, and the edge-guided (EG) image could be expressed as

(2) $$\begin{array}{c} \text{EG}=\sqrt{Ex^{2}+Ey^{2}.} \end{array}$$

*Ex* represented the gradient of the *x*-axis of the image, while *Ey* represented the gradient of the *y*-axis of the image. *Ex* and *Ey* could be expressed as

(3) $$\begin{array}{c} Ex=h∙px, \end{array}$$

(4) $$\begin{array}{c} Ey=h∙py. \end{array}$$

In equations (3) and (4),

(5) $$\begin{array}{c} px=\left[\begin{array}{c} 2\;0-2\\ 2\sqrt{2}\;0\;2\sqrt{2}\;\\ 2\;0-2 \end{array}\right], \end{array}$$

(6) $$\begin{array}{c} py=\left[\begin{array}{c} 2\;2\sqrt{2}\;1\\ 0\;0\;0\;\\ -2-2\sqrt{2}-2. \end{array}\right]. \end{array}$$

The global energy term *F*^*k*^ of the AC model was defined as

(7) $$\begin{array}{c} F^{k}=\kappa_{1}\int {\left|\text{EG}\left(x\right)-k_{1}\right|}^{2}dx+\kappa_{2}\int {\left|\text{EG}\left(x\right)-k_{2}\right|}^{2}dx. \end{array}$$

In equation (7), EG(*x*) represented the value of the *x*th pixel in the EG image, *k*_1_ was the value of the pixel of the EG image within the evolution curve, and *k*_2_ represented the value of the pixel of the EG image outside the evolution curve.

The local energy term *F*^*h*^ of the AC model was defined as

(8) $$\begin{array}{c} F^{h}=\kappa_{1}\int S∙{\left|\text{EG}\left(x\right)-l_{1}\right|}^{2}dx+\kappa_{2}\int S∙{\left|\text{EG}\left(x\right)-l_{2}\right|}^{2}dx. \end{array}$$

In equation (8), *l*_1_ and *l*_2_ were smooth functions, and *S* meant a Gaussian kernel function.

The regularization term *F*^*i*^ of the AC model was defined as

(9) $$\begin{array}{c} F^{i}=\int \frac{{\left|\nabla \varphi \left(x\right)-1\right|}^{2}}{2}dx. \end{array}$$

In the AC model, length constraint term *F*^*j*^ was defined as

(10) $$\begin{array}{c} F^{j}=\int \Omega {\left|\nabla \varphi \left(x\right)\right|}^{2}dx. \end{array}$$

Therefore, the energy functional of the model was updated to be

(11) $$\begin{array}{c} F^{*}=\alpha \kappa_{1}\int {\left|EG\left(x\right)-k_{1}\right|}^{2}dx+\kappa_{2}\int {\left|EG\left(x\right)-k_{2}\right|}^{2}dx+\left(1-\alpha \right)\kappa_{1}\int S∙{\left|EG\left(x\right)-l_{1}\right|}^{2}dx+\kappa_{2}\int S∙{\left|EG\left(x\right)-l_{2}\right|}^{2}dx+\beta \int \frac{{\left|\nabla \varphi \left(x\right)-1\right|}^{2}}{2}dx+\lambda \int \Omega {\left|\nabla \varphi \left(x\right)\right|}^{2}dx. \end{array}$$

Finally, the adaptive image segmentation algorithm PDE-AC under the fourth-order PDE as well as AC model was worked out.

### 2.4. Image Evaluation Indicators and Observation Indicators

The geometric active contour (GAC) model [18] and the advanced modeled iterative reconstruction algorithm (ADMIRE) [19] were introduced to compare with the PDE-AC algorithm in this research. The correct classification ratio (CCR), Dice similarity coefficient (DISC), and average segmentation time (AST) were adopted as the evaluation indicators of image segmentation results. The CCR and DISC were calculated as the following:

(12) $$\begin{array}{c} \text{CCR}=\frac{\left|P\cap Q\right|}{\left|P\right|}, \end{array}$$

(13) $$\begin{array}{c} \text{DISC}=2\times \frac{\left|P\cap Q\right|}{\left|P\right|+\left|Q\right|}. \end{array}$$

In the equations above, *P* represented the segmentation outcome of the PDE-AC algorithm on the image and *Q* represented the segmentation outcome of the gold standard. The basic flow of image processing was shown as Figure 1.

The observation indicators were as follows. The basic information of patients (age, body mass index (BMI), number of male and female cases, hypertension, diabetes, smoking, drinking, triglyceride, total cholesterol, low-density lipoprotein, and high-density lipoprotein) were collected. Serological indicators of patients, including matrix metalloproteinase 7 (MMP7), matrix metalloproteinase 9 (MMP9), and matrix metalloproteinase 12 (MMP12) levels, were counted. These serological indicators were determined using the double-antibody sandwich enzyme-linked immunosorbent assay (ELISA). The OCT images obtained by scanning were sent to the workstation for processing, and related quantitative indicators were measured. Fibrous cap thickness (FCT), lipid plaque length, degree of stenosis, lipid pool angle, macrophages, intimal erosion, plaque fissure, plaque calcification, intraplaque microchannels, and thrombotic conditions were included. The results of CAG were as the gold standard, and the accuracy, sensitivity, and specificity of both OCT images under the PDE-AC algorithm and simple OCT images were calculated.

### 2.5. Statistical Methods

All the data were statistically analyzed using SPSS 19.0. The measurement data were expressed as mean + standard deviation ($\bar{x}\pm s$), while the enumeration data were statistically inferred using *χ*^2^ test. The measurement data conformed to normal distribution, and tested by *t*-test. *P* < 0.05 was considered to be statistically significant.

## 3. Results

### 3.1. Comparison of Segmentation Results of Different Algorithms

As shown in Figure 2, the CCR (0.943 ± 0.105) and DISC (0.985 ± 0.094) of the images segmented and reconstructed by the PDE-AC algorithm were significantly higher than those of the GAC and ADMIRE algorithms, with statistically observable differences (*P* < 0.05). AST (13.482 ± 3.076 ms) of the reconstructed image segmented by the PDE-AC algorithm was statistically lower than that of the GAC algorithm and ADMIRE algorithm (*P* < 0.05).

Figure 3 showed the segmentation and reconstruction results of OCT images by different algorithms. The image quality after processing by the GAC, ADMIRE, and PDE-AC algorithms was improved compared with the original images. In the images processed by the PDE-AC algorithm, artifacts and noise were greatly reduced, and the clarity was also significantly improved. The overall quality was better than the images processed by GAC or ADMIRE.

### 3.2. Comparison of Basic Clinical Data of Patients

Figure 4 displayed the comparisons of the basic clinical data among three groups of patients. Not a statistically significant difference was shown in their age, BMI, number of males and females, hypertension, diabetes, smoking, drinking, triglyceride, total cholesterol, low-density lipoprotein, and high-density lipoprotein in the three groups (*P* > 0.05).

### 3.3. Imaging Manifestations of Cases

As shown in Figure 5, a typical 3-layer structure consisting of the intima, media, and adventitia could be observed in the OCT images of healthy volunteers. The intima was shown as bright bands with high signal, the media showed dark bands with low signal, and the adventitia showed an extracellular matrix and outer elastic lamina. Compared with the OCT images of healthy volunteers, in the OCT images of the patients, the macrophages showed dot-like or strip-like structures of high reflection and strong attenuation, the fibrous cap was intact, and the lumen surface was irregular. The lesions were accompanied by thrombosis, with no superficial lipid and calcification in the proximal or distal to the thrombus.

### 3.4. Comparison of Serological Indicators

In Figure 6, there was not a significant difference in the level of MMP12 among the three groups of patients (*P* > 0.05). The levels of MMP7 and MMP9 in the unstable plaque group were remarkably higher than those in the stable plaque group and control group; the differences were of statistical significance (*P* < 0.05). The levels of MMP7 and MMP9 were not statistically different between the stable plaque group and control group (*P* > 0.05).

### 3.5. Comparison of OCT Quantitative Indicators between Stable Plaque Group and Unstable Plaque Group

As presented in Figure 7, there was no remarkable difference in plaque calcification, intraplaque microchannels, and thrombus between the stable plaque group and the unstable plaque group (*P* > 0.05). Lipid plaque length, degree of stenosis, and lipid pool angle, macrophages and intimal erosion, and plaque fissure in the unstable plaque group were considerably greater than those in the stable plaque group, with the differences of statistical significance (*P* < 0.05). The FCT of the unstable plaque patients was significantly smaller than that in the stable plaque group, showing a statistically significant difference (*P* < 0.05).

### 3.6. Comparison of Diagnostic Effect between OCT Images under PDE-AC Algorithm and Simple OCT Images

In Figure 8, the diagnostic sensitivity of OCT images under the PDE-AC algorithm for CHD was 91.53%, the diagnostic specificity was 84.08%, and the diagnostic accuracy was 95.38%. The diagnostic sensitivity, specificity, and accuracy of the simple OCT images for CHD were 83.46%, 75.11%, and 88.02%, respectively. The diagnostic sensitivity, specificity, and accuracy of OCT images under the PDE-AC algorithm were all markedly higher than those of simple OCT images with differences of statistical significance (*P* < 0.05).

## 4. Discussion

The gold standard for clinical diagnosis of CHD is CAG. CAG is an interventional examination that can intuitively reflect the stenosis of cardiac vessels. It is currently the most reliable method for diagnosing CHD. However, the invasiveness of CAG to patients limits its development, and it is necessary to seek more scientific diagnostic methods [20, 21]. Thus, 82 CHD patients who were going to undergo CAG for confirming the condition were included in this research as the research objects. According to the CASS diagnostic criteria for CHD, the patients were divided into the stable plaque group with 41 cases and the unstable plaque group with the other 41 cases. Furthermore, 20 healthy volunteers having physical examination during the same period were chosen as the control group, and all the patients as well as volunteers underwent OCT. For the improvement of quality of OCT images, the fourth-order PDE and AC model were also introduced in this research, to construct a novel adaptive image segmentation algorithm PDE-AC. The PDE-AC algorithm was then compared with the GAC algorithm and ADMIRE algorithm. The GAC algorithm is on the basis of the methods of curve evolution and level set. It implicitly expresses the two-dimensional evolution curve as a three-dimensional continuous function and follows certain rules to continuously update the level set function. Thus, the implicit closed curve can be evolved [22]. ADMIRE is a third-generation MRI technology that compares the virtual raw data generated by forward projection with the projection data actually collected by the detector for multiple times, to eliminate artifacts and reduce noise [23]. The CCR (0.943 ± 0.105) and DISC (0.985 ± 0.094) of the segmented and reconstructed images by the PDE-AC algorithm were statistically higher than those of the GAC and ADMIRE algorithms (*P* < 0.05). Such a result was similar to the findings of Gu et al. [24], indicating that the PDE-AC algorithm proposed in this research was better than the traditional algorithm for segmentation of OCT images. Thus, the PDE-AC algorithm had a certain clinical application value. In addition, the AST (13.482 ± 3.076 ms) of the reconstructed image segmented by the PDE-AC algorithm was statistically and significantly lower than that of GAC and ADMIRE (*P* < 0.05). Compared with PDE-AC, the shortcomings of the other two algorithms were also quite obvious. For example, the constant evolution speed needed to be manually determined according to the position of the initial curve, adaptive segmentation could not be achieved, and boundary leakage was prone to occur. While the PDE-AC algorithm could achieve adaptive segmentation, and the evolution speed changed with the position of the evolution curve, which avoided boundary leakage to a certain extent and had a better performance.

In this research, the basic clinical data of three groups of patients were first compared. None of statistically significant difference was discovered in the pairwise comparisons of their age, BMI, number of males and females, hypertension, diabetes, smoking, drinking, triglyceride, total cholesterol, low-density lipoprotein, and high-density lipoprotein (*P* > 0.05). This result provided feasibility for follow-up study. Then, the quantitative data indicators of OCT of the patients were compared. The lipid plaque length, degree of stenosis, lipid pool angle, macrophages, intimal erosion, and plaque fissure of the unstable plaque group were statistically markedly greater than those of the stable plaque group, while FCT was statistically thinner (*P* < 0.05). Thereout, it was indicated that the lipid plaque length, the degree of stenosis, the angle of lipid pool, macrophages and intimal erosion, plaque fissure, and FCT were important indicators for interpreting the presence of unstable plaques [25, 26]. With micron-scale axial resolution, OCT could accurately determine FCT and the cellular composition of the fibrous cap in vulnerable plaques formed by lipids on the vessel wall. It was also more sensitive in detecting thrombi and dissections. The image features of OCT scans could determine the stability of plaques in patients with CHD and help physicians to assess the progress of the disease timely. Specificity and accuracy of OCT images under PDE-AC algorithm for diagnosing CHD were statistically and significantly higher than those of simple OCT images (*P* < 0.05). This further revealed that the PDE-AC algorithm-based OCT images were superior to simple OCT images in the diagnosis of CHD, deserving a better clinical application value.

## 5. Conclusion

In this research, OCT scans were performed on all three groups of objects, and the images were segmented by the PDE-AC adaptive algorithm. The PDE-AC algorithm not only showed excellent image segmentation effect but also had high operating efficiency and good comprehensive performance. OCT images under the PDE-AC algorithm were better than simple OCT images in the diagnosis of CHD. Lipid plaque length, degree of stenosis, lipid pool angle, macrophage and intimal erosion, plaque fissure, and FCT were important indicators for judging plaque stability, having the better clinical application value. However, due to time and budget constraints, this research included a small size of samples from a single source. Meanwhile, in view of safety, acute myocardial infarction cases were not included, so there was a certain selection bias. Reinclusion of CHD patient samples would be considered in the future, to further analyze the application value of OCT images under the PDE-AC algorithm. In conclusion, this research gave a reference for the imaging diagnosis of clinical CHD.

## Figures and Tables

**Figure 1:** Image processing process under PDE-AC.

**Figure 2:** Comparison of segmentation outcome indicators under different algorithms. (a–c) CCR, DISC, and AST, respectively. ^∗^Compared with PDE-AC algorithm, *P* < 0.05.

**Figure 3:** Segmentation and reconstruction outcomes of OCT images by different algorithms. (a) The original image. (b) Under GAC algorithm. (c) Under ADMIRE algorithm. (d) Under PDE-AC algorithm. The green area in the picture is a calcified plaque.

**Figure 4:** Comparison of basic data of three groups of patients. (a) Age and BMI. (b) The number of male and female cases. (c) Hypertension and diabetes. (d) Smoking and drinking. (e) Triglycerides and total cholesterol. (f) Low-density lipoprotein and high-density lipoprotein.

**Figure 5:** Imaging manifestations of the cases. Male patient, 67-year-old, with unstable angina pectoris. (a) OCT image of a healthy volunteer. (b–d) OCT images.

**Figure 6:** Comparison of serological indicators among three groups. (a–c) MMP7, MMP9, and MMP12, respectively. ^∗^Compared with the levels in the unstable plaque group, *P* < 0.05.

**Figure 7:** Comparison of lesion volume between the two groups before and after treatment. (a) FCT and the lipid plaque length. (b) Degree of stenosis and the angle of the lipid pool. (c) Macrophages and intimal erosion. (d) Plaque fissure and plaque calcification. (e) Comparison in intraplaque microchannel and thrombus. ^∗^Compared with the stable plaque group, *P* < 0.05.

**Figure 8:** Comparison of the diagnostic effect between the PDE-AC algorithm-based OCT images and simple OCT images. ^∗^Compared with origin OCT images, *P* < 0.05.

## Data Availability

The data used to support the findings of this study are available from the corresponding author upon request.
